# Peculiarities of Integrating Mechanical Valves in Microfluidic Channels Using Direct Laser Writing

**DOI:** 10.1155/2022/9411024

**Published:** 2022-10-07

**Authors:** Lucero Hernandez-Cedillo, Deividas Andriukaitis, Lukas Šerpytis, Tomas Drevinskas, Olga Kornyšova, Vilma Kaškonienė, Mantas Stankevičius, Kristina Bimbiraitė-Survilienė, Audrius Sigitas Maruška, Linas Jonušauskas

**Affiliations:** ^1^Laser Research Center, Vilnius University, Saulėtekio Ave. 10, Vilnius LT-10223, Lithuania; ^2^Femtika, Saulėtekio Ave. 15, Vilnius LT-10224, Lithuania; ^3^Institute of Chemistry, Vilnius University, Naugarduko 24, 03225 Vilnius, Lithuania; ^4^Instrumental Analysis Open Access Centre, Vytautas Magnus University, Vileikos 8, Kaunas LT-44404, Lithuania

## Abstract

Regenerative medicine is a fast expanding scientific topic. One of the main areas of development directions in this field is the usage of additive manufacturing to fabricate functional components that would be later integrated directly into the human body. One such structure could be a microfluidic valve which could replace its biological counterpart in veins as it is worn out over the lifetime of a patient. In this work, we explore the possibility to produce such a structure by using multiphoton polymerization (MPP). This technology allows the creation of 3D structures on a micro- and nanometric scale. In this work, the fabrication of microfluidic systems by direct laser writing was carried out. These devices consist of a 100 *μ*m diameter channel and within it a 200 *μ*m long three-dimensional one-way mechanical valve. The idea of this device is to have a single flow direction for a fluid. For testing purposes, the valve was integrated into a femtosecond laser-made glass microfluidic system. Such a system acts as a platform for testing such small and delicate devices. Measurements of the dimensions of the device within such a testing platform were taken and the repeatability of this process was analyzed. The capability to use it for flow direction control is measured. Possible implications to the field of regenerative medicine are discussed.

## 1. Introduction

Additive manufacturing brought a lot of advances to various fields [1]. Regenerative medicine is one of them [2]. So far, various structures for medical research and implantation were produced using three-dimensional (3D) printing. One of the most interesting prospects is the usage of femtosecond (fs) laser-based multiphoton polymerization (MPP) to produce structures for biomedical use [3]. So far, main progress was achieved with various scaffolds for cell research [4], cultivation [5], and implantation [6]. However, as evident from other types of 3D printing, more complex structures could be produced. One type of such structure is valve [7]. Indeed, these can find many uses in medicine, the most exotic being direct biovalve replacement in the cardiovascular system [8]. While standard 3D printing can produce such structures at the heart scale, MPP could be used to print smaller, vein-level objects [9].

While theoretically MPP-produced structures look very promising, one of the key challenges with them is testing. Indeed, when structures become submillimeter, their handling becomes very difficult. The reason for it is both very small scale requiring very precise tools as well as inherent brittleness of these devices. This means that adapting existing testing infrastructure for testing at the microscale becomes highly nontrivial. However, fs pulses used in MPP can also be used in much different processing regimes [10]. As was shown before, single fs direct laser writing (DLW) setup, consisting of a laser, positioning system, and optical chain, can be used for both subtractive and additive manufacturing in subsequent steps [11–13]. As a result, one way to potentially simplify MPP-made structure testing is to potentially integrate them in some other, bigger laser-made substrates, such as for instance, microchannels. As these are normally made out of more robust materials like glass [14], they can be handled more easily. Also, such objects can be made to fit more standard devices available in testing facilities, like pumps. Thus, it means that using fs DLW can yield both highly precise functional structure made using additive MPP and a platform for its testing made by subtractive fs DLW means.

This work is dedicated to testing the concept of using hybrid subtractive-additive fs DLW to produce both highly precise functional 3D structure and its testing platform. We chose a ball valve as a model structure and will integrate it into a custom-tailored glass channel for testing. While MPP is capable of producing more complicated valve designs [9, 15], the ball valve is much simpler and compact as it does not require a return spring, which would put additional emphasis on the mechanical properties of the polymer. We provide considerations needed for such an operation. Valves are characterized both from geometry and functionality standpoints, providing insight into how testing in microfluidic channels might have influenced it. Also, general insight into manufacturing peculiarities and how they can influence the function of the valve is provided.

## 2. Methods and Materials

Following the schematics in Figure 1, the manufacturing process of these devices can be divided into two main parts of DLW. The first part is to make the microchannel in the glass and the second part is to create the microvalve inside the channel. All of this was carried out using the “Laser Nanofactory” (Femtika) setup. It was either tuned for subtractive manufacturing by applying an F-theta lens or used for additive manufacturing by employing an immersion microscope objective (63 × 1.4 numerical aperture (NA) by Zeiss). The soda-lime glass was used as a channel material. SZ2080 was chosen as a prepolymer as it exhibits minimal shrinkage [16] and has well predictable mechanical properties [17]. A drop of prepolymer doped with 1% of photo-initiator Irgacure 369 (IRG for short) was added to the cover glass (for isolated valve fabrication) or channels and left at 50°C overnight to prebake. After laser printing, the structure is exposed to methyl isobutyl ketone for 5 min to reveal it. Such a short development time is allowed by a very small amount of prepolymer in the channel. Also, it allows for avoiding excessive swelling during development [18], which can damage the final device. In this work, the valves were observed under an optical microscope and their measurements were taken to see how reproducible is the method. More information on setup and polymerization parameters can be found in our previous work [19]. Parameters and considerations used for channel cutting are described in a dedicated research study by our group [13].

Additional note about the integration of polymeric structures into glass channels using MPP. Normally, during MPP, cover glass with polymer drop on it is used. If an immersion objective is employed (like in this work) for fabrication and the prepolymer is liquid, the dip-in technique [20] or working distance expander [21] can be used for fabrication. However, this cannot be done with hard prepolymers, like SZ2080 or SU8, which can also be processed quite easily using MPP [22]. Then, immersion oil is put on the other side of the cover glass, and fabrication is carried out with prepolymer drop-down. Challenge in this work was that polymer structures had to be integrated into a channel. In other previous studies, prepolymers are introduced into the channel, prebacked, and laser exposure is done inside the closed channel [11, 12]. However, in this work, fs laser was used to ablate the open channel, which subsequently was sealed using thermoplastic. Thermoplastic dissolves in the standard SZ2080 developer; thus, fabrication has to be done with an immersion objective in the open channel using the hard prepolymer. The solution to this issue is to apply immersion oil directly on the prepolymer drop [Figure 2]. Then, the immersion objective can be used even with a hard prepolymer. While in this work this was applied to integrate polymer structures into glass channels, this can also be employed to win some of the working distance of immersion objectives, as instead of focusing through cover glass all of that thickness translates to an overall fabricated structure height. After, the fabrication immersion oil is dissolved by the same developer which is used for the prepolymer. Nonetheless, care should be taken when operating in such an arrangement, as the prepolymer drop height should not exceed the working distance of the objective. If this happens, there is a chance that the exit aperture of the objective will touch the hard prepolymer drop top, subsequently damaging it. This is the main limitation of this approach. Also, some immersion oils have additives in them, which slowly dissolve some of the prepolymers. Appropriate, solvent-free immersion oils should be used to avoid it completely, or the fabrication time should be kept to a minimum (no more than a few hours). Also, the immersion objective should be cleaned after each such experiment to avoid long-term contamination by the dissolved prepolymer.

## 3. Results

We began our work by fabricating a valve on the glass substrate. The goal was to see if such a structure can be produced using the standard manufacturing mode. The outer architecture of the valve was chosen to be square to accommodate further integration into the microfluidic testing platform. Nevertheless, for biological applications, round, tubular architecture can be employed. As we can see from Figure 3(b), manufacturing on glass yielded a nearly perfect valve. The ball was free-floating, showing that by using SZ2080 prepolymer, which is a hard gel during the printing process, free, unattached elements can be produced. This is a huge advantage in comparison to most other 3D printing techniques, which would require support for such elements as a ball inside valve [23]. While in macro 3D printing, these can be easily removed; in micro-case, it would be nearly impossible.

Furthermore, the valve was integrated into a glass channel, in which it will be tested. Glass channels were 120 *μ*m wide and 100 *μ*m deep and made out of soda-lime glass. Inlets and outlets were 1 mm diameters. As with all additive integration of structures into other geometries, aligning sample rotation and depth were the most important considerations. Luckily, MPP setups have integrated imaging systems allowing us to very precisely gauge these parameters [24]. They can then be used in the software controlling the setup to compensate the model for the printing process. Indeed, a rotating 3D model is a lot easier than the rotating channel system as it would require additional rotational axes, which would add to the price of the setup. After compensation is performed, the valve can be easily integrated into the channel [Figure 3(e)]. Overall, 10 such systems were produced and tested.

One important parameter when considering real-world applications of additively produced 3D structures is the repeatability of dimensions. Indeed, keeping in mind the extremely strict requirements of medical device manufacturing, any deviations should be minimal. Thus, key components of the device have to be tested. The valve consists of a structure with a sphere inside and at one of the entrances a circular hole and the other scaffolding to prevent the sphere from escaping. The circular hole stops the sphere; the idea is that the sphere matches the hole so as not to let it escape and in turn prevent the passage of the flow. Measurements of the critical components of the valve inside the channel are shown in Figure 4. In the graph, the place where the measurement was taken is related by color and number. The square area shows the general dispersion of measurements with statistical errors being shown from the average value. The color-coded areas are as follows: in light green is the width of the structure and dark blue denotes the length of the valves. Red denotes a longitudinal beam that prevents the sphere from escaping from the structure during its development and before sealing the device. Light blue shows the thickness of the surface stopping the ball from escaping during pressurized operation. These four parameters showed great repeatability, with the deviation of measurement being close to ∼1–2%. This is to be expected, as the material used, SZ2080, was created as a ultralow shrinkage material [16]. Subsequently, the deviation from the model dimensions was also around or below 1–2%. Also, it should be noted that all these measurements are taken in the horizontal direction.

Deviation in other parts of the device is substantially higher. In purple are the walls of the valve. Their deviation reaches ∼23%. This can be explained by their close proximity to the supporting channel walls. As channel walls can have significant deviations because of the fast cutting method [13], this translates to the valve walls being either deformed outward during fabrication or becoming seemingly thinner due to being partially inside the glass wall. However, as these only support structures, their deviations do not play an important role in the functionality of the device and seemingly would be much closer to the desired dimensions in the final device where channel walls are not present.

Next, in pink, we have the diameter of the sphere. The deviation of this component is in the range of ∼4.5%. While seemingly not much, the ball is the main functional component and its precision is crucially for the appropriate functionality of the device. Furthermore, the component in which the ball should sit during operation, the main opening, has a size deviation of 10.9%. Therefore, in effect, it means that the two main components of such valves have inherently the highest deviation in the most crucial parts. The reasons for it can be a combination of general structure shrinkage as well as aberrations occurring during printing. The latter is quite evident because of quite a high deviation of the overall valve height from sample to sample (dark green). Indeed, as a high NA (1.4) objective was used for printing, the laser light has to pass immersion oil, then the surface of the prepolymer (which is, by the way, slightly curved due to meniscus which forms when prepolymer is deposited), and then it has to pass a somewhat varied thickness of the drop (as each polymer drop is slightly different). While immersion oil and SZ2080 should have relatively similar refractive indexes, their deviation is still sufficient to cause some focusing abnormalities at such high NA [25]. This also explains why features that have critical sizes in a horizontal direction have minimal deviations. Luckily, if this would prove to be detrimental to the functionality of such a device, a spatial light modulator (SLM) can be used to dynamically correct it during printing [26, 27].

Among repeatability deviations, generally printing within glass channels has other risks. Alignment problems not only create an asymmetric structure, but this asymmetry also makes structures less rigid and can break at the time of development or during handling. In Figure 5, we can see a functional valve in the center and on the right a valve that was printed with an inappropriate alignment of the channel with the laser. In this last condition, we can observe that the retention structures at the ends of the valve can fragment and leave the valve inoperable. This is further compounded if the development is longer than several minutes. It not only increases the probability of structure breaking but also can lead to polymer device delaminating from the channel, rendering it completely inoperable. However, these defects are not very common (less than 1 fabrication out of 10) and can be easily avoided if proper alignment and development procedure is employed.

Finally, the devices were tested with water to see if they operate as a one-way valve. The flow rate was varied between 0.5–3 ml/min. The microfluidic pump has a pressure sensor that indicates if the flow is being obstructed, the higher the pressure the less flow is passing through the microfluidic device. These experiments were carried out in two configurations, in valve mode, with the flow in the direction of the valve that prevents the passage of water, and in normal mode, with the flow in the direction where the water can pass. In Figure 6, it can be seen that in valve mode, the pressure is at least twice the pressure in normal mode. Therefore, despite all the listed difficulties and deviations, valves fundamentally work. Nevertheless, further optimization, especially for consistent ball and hole size, is needed to achieve more consistent operation as well as higher blockage of liquid in valve configuration.

## 4. Discussion

MPP usage in biomedical applications is rising steadily. It is motivated by design freedom and a huge selection of suitable materials [28, 29], including biopolymers [3]. Also, as MPP is an additive manufacturing technique, designs for medical structures can be tuned very easily, creating excellent synergy with patient-specific personalized medicine [30]. However, so far, it was shown primarily as a technology to produce scaffolds for cell cultivation, investigation, or possible implantation. However, despite it, there are other ways of using MPP, especially for devices that have some movable parts [19, 31]. As shown in this work, MPP can be used for more advanced structures, such as micro-valves [9, 15] which could replace worn-out ones in the cardiovascular system. This would greatly supplement the current progress of 3D-printed cardiovascular systems already being shown in various literature.

However, working on such a scale brings both new capabilities and challenges. Testing of such devices might be difficult both due to their size and brittle nature. As we showed here at least some testing can be done by integrating prototypes into prefabricated, robust microfluidic systems. This allows us to uncover some initial nuances of the devices, like potential size deviations due to material shrinkage and aberrations observed in this work. Another option would be to use glass micromechanics, produced by fs selective glass etching (SLE). These were shown to also provide assembly-free capabilities of fabrication, somewhat similar to MPP, yet more sensitive to manufacturing parameters [32]. Additionally, multistep 3D additive manufacturing can also be employed in a similar fashion [33–35]. However, while glass or other inorganic materials can be used for initial testing, it is a hard material and does not well represent the mechanical properties of live tissue [36–38]. Thus, a compromise between ease of testing, mechanical properties of the final structure, and design optimization needs to be found.

## 5. Conclusions

In this work, we use fs DLW to produce a high-precision 3D ball valve inside a glass microchannel testing platform. We show that valve design can be easily adopted for such applications. Generally, fabrication was proven to be satisfactory, with features in horizontal dimensions being within a 1–2% deviation from the intended size. The noticeable exception are side walls, which were deformed due to close proximity to channel walls. This shows that some care should be taken when considering MPP 3D structure integration into glass channels. Also, unrelated to the integration peculiarities, all structural components made in vertical directions showed significant size deviation, sometimes exceeding 20%. This was speculated to be a result of aberrations occurring during laser exposure. Despite it, the general functionality of a valve was observed, providing that the design is sound and could be used in the future after some precise tuning.

## Figures and Tables

**Figure 1:** Simplified diagram of the manufacturing process. In the upper part, the laser writing process of the microchannel in glass. In the lower part, the laser writing of the valve inside the channel.

**Figure 2:** Steps of integrating the polymeric structure into an open glass channel using the hard prepolymer (in our case SZ2080) and immersion objective. (a) Prebake of the material. (b) Integration of functional element into the channel by applying immersion oil onto hard prepolymer. (c) Development. (d) Finished structure.

**Figure 3:** (a) 3D model of the valve used for fabrication. (b) and (c) Optical image and SEM micrograph of valve on the glass substrate. No deviations from the planned geometry can be detected. (d) 3D model of the valve inside the channel. (e) Integrated polymeric 3D valve inside the glass channel.

**Figure 4:** Measurements of different sections of the valve were recorded inside the microchannels.

**Figure 5:** On the right - STL model and structures manufactured within the micrometric channels. In the center is an ideal structure. On the right are the possible manufacturing errors.

**Figure 6:** Flow experiment. The devices were tested in both directions, valve mode and normal mode, at different flow rates of 0.5, 1, 1.5, 2, 2.5, and 3 ml/min to verify the operation of the one-way valve.

## Data Availability

Data underlying the results presented in this study are not publicly available at this time but may be obtained from the authors upon reasonable request.
